# A comparative study of the policy response to COVID-19 in the ASEAN region: A dynamic simulated ARDL approach

This article has been retracted.

**DOI:** 10.1371/journal.pone.0276973

**Published:** 2023-01-26

**Authors:** Nihal Ahmed, Dilawar Khan, Judit Oláh, József Popp

**Affiliations:** 1 Department of Economics, Kohat University of Science and Technology, Kohat, Pakistan; 2 Department of Management, Faculty of Applied Sciences, WSB University, Dabrowa Górnicza, Poland; 3 Hungarian National Bank–Research Center, John von Neumann University, Kecskemét, Hungary; 4 College of Business and Economics, University of Johannesburg, Johannesburg, South Africa; Bucharest University of Economic Studies: Academia de Studii Economice din Bucuresti, ROMANIA

## Abstract

The COVID-19 epidemic is the most significant global health disaster of this century and the greatest challenge to humanity since World War II. One of the most important research issues is to determine the effectiveness of measures implemented worldwide to control the spread of the corona virus. A dynamic simulated Autoregressive-Distributed Lag (ARDL) approach was adopted to analyze the policy response to COVID-19 in the ASEAN region using data from February 1, 2020, to November 8, 2021. The results of unit root concluded that the dependent variable is integrated of order one while the independent variables are stationarized at the level or first difference, and the use of a dynamic simulated ARDL technique is appropriate for this paper. The outcomes of the dynamic simulated ARDL model explored that government economic support and debt/contract relief for poor families is substantially important in the fight against COVID-19. The study also explored that closing schools and workplaces, restrictions on gatherings, cancellation of public events, stay at home, closing public transport, restrictions on domestic and international travel are necessary to reduce the spread of COVID-19. Finally, this study explored that public awareness campaigns, testing policy and social distancing significantly decrease the spread of COVID-19. Policy implications such as economic support from the government to help poor families, closing schools and public gatherings during the pandemic, public awareness among the masses, and testing policies must be adopted to reduce the spread of COVID-19. Moreover, the reduction in mortality shows that immunization could be a possible new strategy to combat COVID-19, but the factors responsible for the acceptability of the vaccine must be addressed immediately through public health policies.

## Introduction

Epidemics are biological calamities that arise because of the wide spread of infectious diseases that are usually produced by viruses, parasites, and viruses. These are the most shocking of all-natural calamities for which humanity is suffered. Understanding earlier epidemics is crucial for controlling and preventing future epidemics [1]. History reveals frequent pandemics, including SARS-CoV in 2003 [2], Influenza A (H1N1) in 2009 [3], Middle East respiratory syndrome (MERS-Cov2) originating in 2012 [4]. The Polio pandemic appeared in 2014, Zika in 2016 and Ebola in the Democratic Republic of Congo in 2019. The current COVID-19 pandemic is regarded as the most critical global health disaster of the era, as well as the biggest threat to mankind since World War II. The problem spread quickly across the world, posing significant social and economic challenges to human health [5]. It affected more than 250,056,541 people and killed more than 5,052,620 people worldwide. These numbers are increasing rapidly. This pandemic also affected ASEAN countries and affected more than 12,640,210 people and killed more than 266,203 people in this region. The World Health Organization (WHO) also declared the outburst of COVID 19 as the 6^th^ Emergency Public Health Service (SPHEC) on January 30, 2020 [6].

COVID-19 first appeared in Wuhan, in the province of Hubei, China. Its medical symptoms were closer to viral pneumonia. The WHO later declared this outbreak as a public health emergency of international alarm on January 30, 2020 [7]. To reduce the suspected cases and fatalities of COVID-19, governments have imposed several containment measures, including school closures, border closures, quarantine and isolation, restrictions on public transport and air travel in countries that make up the world’s largest economies. This is raising the fear of an economic slowdown and an abrupt recession [8].

Health professionals, governments and the public need unanimity and fight shoulder to shoulder to control this pandemic [9]. In addition to the widespread spread of the corona virus, precautionary actions have also added toward the global economic downturn [10]. In addition, several governments have adopted different measures and the speed with which they have been adopted. This disparity gave rise to a discourse on how policymakers and the public would plan the level of response to these preventive measures. This forces them to implement or retreat from these measures. Once death-related events happen, it is essential for the companies to offer sufficient directives to workers rather than ignore them [11]. The public health specialist learns in real time the strategies if they are effective or not [12]. (Fig 1) gives government policies to lessen the risk of dissemination of COVID-19.

**Fig 1:** Government policies to reduce the risk of dissemination of COVID-19.

The rapid dispersion of the new coronavirus accredited primarily to the increased percentage of unreported infections [13] makes pandemic control more challenging. Finally, notable, and unusual public health measures have been adopted by most economies, imposing inflexible initiatives at the national levels to impede the virus’s spread in their countries. The decline in man-made activities has had a positive influence on the natural environment [1, 14]. The COVID-19 epidemic arises in China and has spread to ASEAN countries in a few months. The pandemic is more exciting and threatening for ASEAN countries, as these countries are socially, economically, and geographically different from each other [15]. One of the theories about why Asian countries like Cambodia, Laos, Myanmar, Thailand and Vietnam have comparatively fewer cases of COVID-19 losses is because of their cultural perspective [16]. (Fig 2) shows **c**omparison of COVID-19 confirmed cases in ASEAN countries. Moreover, (Fig 3) Shows COVID-19 death cases in ASEAN countries.

**Fig 2:** COVID-19 confirmed cases per million population in ASEAN countries [20].

**Fig 3:** COVID-19 death cases per million population in ASEAN countries [20].

The main reason for COVID-19 cases imported into ASEAN countries is foreign workers and migration [17]. Economies are classified as transfer countries (Cambodia, Indonesia, Laos, Myanmar and Philippines) and as receipt countries (Brunei, Thailand, Malaysia and Singapore). Singapore and Vietnam mixed during the COVID-19 epidemic, applying various precautionary strategies, including testing, screening, and screening method [18]. Table 1 shows COVID—19 first case registered in ASEAN countries.

**Table 1:** COVID—19 first case registered in ASEAN countries.

S.no.	Country	COVID–19 date of 1^st^ registered case
1	Brunei	Mar 09, 2020
2	Cambodia	Jan 31, 2020
3	Indonesia	Mar 02, 2020
4	Laos	Mar 24, 2020
5	Malaysia	Jan 25, 2020
6	Myanmar	Mar 23, 2020
7	Philippines	Jan 30, 2020
8	Singapore	Jan 23, 2020
9	Thailand	Jan 22, 2020
10	Vietnam	Jan 23, 2020

Source: World Health Organization (2020)

ASEAN countries have made progress in vaccinating their populations despite capacity issues in their health systems. There are no previous health initiatives that are comparable to the COVID-19 vaccination campaign, so a look at regional health systems may not be a fair predictor of how immunizations will be delivered. Herd immunity initiatives face difficulties in gaining adequate acceptance of vaccinations. A take-up rate of 77.7 percent is required for a vaccination that is 90 percent effective in reaching the herd immunity threshold of 70 percent in a population. The average take-up in the region is 64%. According to a study undertaken in collaboration with Facebook, the World Health Organization, Massachusetts Institute of Technology, and Johns Hopkins University, the region’s acceptance rate is high compared to North America 50% and low in compared to China’s estimated acceptance rate of 84 percent [13]. Numerous studies have established a significant correlation between education and family socioeconomic status and the likelihood of immunization [19]. (Fig 4) provides the COVID-19 vaccination acceptance rate for the region.

**Fig 4:** Willing to accept COVID-19 vaccination in ASEAN countries. Source: COVID-19 Beliefs, Behaviors & Norms Survey (2021).

It is estimated that 50.9 percent of the world population has already been vaccinated (at least one dose) against the coronavirus. More than 7.25 billion doses have been administered worldwide, and 27.23 million doses are administered daily. It is also estimated that only 4.1 percent populations in low-income region has received at least one dosage of vaccination. Table 2 provides a summary of the vaccination statistics for ASEAN countries as of November 2021 [20].

**Table 2:** Summary of vaccination statistics.

Country	Vaccination administered	Fully vaccinated population	Fully vaccinated (% of population)
Brunei	626,279	272,318	62.84%
Cambodia	27,910,923	13,123,236	79.59%
Indonesia	204,233,413	78,114,072	28.86%
Laos	4,402,770	2,776,646	38.72%
Malaysia	50,462,307	24,625,458	77.07%
Myanmar	20,034,000	6,966,000	12.9%
Philippines	62,474,334	33,755,478	31.22%
Singapore	10,094,499	4,703,751	82.47%
Thailand	79,517,972	32,726,021	47.00%
Vietnam	86,319,808	26,964,109	27.95%

Data source: Johns Hopkins Coronavirus Resource Center

The COVID-19 pandemic has severely affected different sectors across the world. It also created major challenges for the ASEAN region. Several measures are being taken in countries in this region to reduce the severity of this pandemic. These measures include economic support, stringent, and health and containment measures. This study employed a dynamic simulated Autoregressive-Distributed Lag (ARDL) approach. Based on study’s findings, policymakers in these nations will be better able to reduce the spread of the COVID-19 infection. Moreover, the article will provide an insight into which ASEAN countries are coping better with the COVID-19 problem. In this way, these countries will be able to benefit from each other’s experiences to effectively manage the corona virus. The results of the study would be a decision-making guide for policymakers to combat pandemics and future disasters as well. The results would also be applicable internationally that would cooperate all territories to go through such a critical situation and regulate the prevalence of contagion.

This study has the following objectives (a) to assess the effect of policy measures adopted by ASEAN countries to control the COVID -19 pandemic (b) to comparatively analyze the policy steps of ASEAN countries to the reduction of the COVID-19 infection. Moreover, this research will test the following hypotheses both in the short and long runs: (a). The economic support for the poor provided by the countries significantly reduces the spread of the COVID-19 infection (b). The stringency measures such as workplace closures, school closures, closures of public transport, restriction on public gathering, public information campaign, stay-at-home, restrictions on internal transport and international travel restrictions significantly reduce the spread of COVID-19 pandemic (c). Containment and health steps such as testing policy, contact tracing, face covering, vaccination policy and number of people vaccinated play a significant role to curb COVID-19 epidemic.

The rest of this paper is structured as follows: The second section examines the literature review; the third section explains the study’s methodology; the fourth section discusses the study’s outcomes, and the final part analyzes the study’s conclusions and policy prescriptions.

### Literature review

This section covers the review of literature directly or indirectly related to this study. COVID-19 is a worldwide pandemic and has severely influenced the global economy [21]. It also presented challenges for the ASEAN region due to its huge population, poor socioeconomic conditions, high poverty and poor health facilities. Most previous studies conducted on the COVID-19 pandemic are theoretical in nature and not directly related to this study. These are summarized as below:

Clark et al. [22] evaluated the effect of coronavirus disease in 2019 on African and ASEAN health systems and national resources. They found that 349 million people 4% of the world population are at huge risk of COVID-19 pandemic. Loomba, de Figueiredo [23] conducted a study to measure the influence of COVID-19 vaccine misinformation on vaccination intent in the United Kingdom and United States. The study found that scientific misinformation is significantly correlated with decline in vaccination intention. Barbera, Jones [24] employed financial “Resilience” to discover the capabilities of governments to absorb, anticipate and response to shocks and calamities in the framework of local governments in Austria, England and Italy. Klimanov, Kazakova [25] tried to develop government financial resilience in emerging economy contexts in Russia. Atkeson [26] conducted a study in United States and investigate the economic influence of COVID-19 in the region. The study found a relationship between the severity and timing of disease suppression through disease progression and social distancing in the population. Sarihasan, Oláh [27] discovered that in high-reliability healthcare companies, shared knowledge patterns, self-care, and awareness of corona infection repercussions at work have a larger role in preventing Covid-19. Khan et al. [42] explored the impact of policy pleasured taken by the South Asian region to curb the COVID-19 infection employing panel data. They found that the policies taken by these countries significantly reduce the COVID-19 pandemic.

Keeping in view the above literature, the research gaps that this paper fills are twofold: first, most studies carried out in the past in these countries or in other areas of the world are primarily theoretical in nature. Findings based on the actual data collected are more reliable and differentiated. Many national and international organizations have compiled data on the COVID-19 pandemic and its preventive measures for every country in the world. Thus, the results of this study are based on recent data collected from different international organizations. Finally, this study comparatively analyzes the effectiveness of different preventive measures against COVID-19, including economic support, stringent, and health and containment measures adopted by the ASEAN region to decrease the rapid spread of the COVID-19 infection in contrast to some studies conducted as a cluster in another region.

## Methodology

The main aim of this study is to comparatively analyze the policy response to the reduction of the COVID-19 pandemic in the ASEAN region. The nature of this research is based on weekly time series data for the period Feb 2, 2020, to November 8, 2021, for the ASEAN countries. This region includes Brunei, Cambodia, Indonesia, Laos, Malaysia, Myanmar, Philippines, Singapore, Thailand, and Vietnam. Government around the world have taken several responses to reduce the impact of the COVID-19 pandemic including economic support, stringency, and containment and health measures. Therefore, this study uses four indices which are the COVID-19 index (CO), the economic support (ES) index, the stringency index (SI), and the Containment and Health (CH) index. The three indices were taken from the Oxford Coronavirus Government Response Tracker [28–30]. The weekly COVID index was composed by the following formula [31]:

$$COVID\;19\;Index=Ln(1+R_{it}+D_{it})$$ (1)

Here *Ln* gives the natural logarithm, *R*_*it*_ represents the number of cases taken at time *t*, and *i* refers to each country. *D*_*it*_ depicts the number of death cases at time *t*, *i* is for each country. The weekly COVID index is treated as a dependent variable. In addition, the independent variables include economic support (ES) index, the stringency index (SI), and the Containment and health index (CH) are used to capture the effect of these measures in decreasing COVID-19 in ASEAN countries. The author describes the variables in Table 3. Fig 5 shows the flowchart of methodology.

**Fig 5:** Flowchart of the methodology.

**Table 3:** Description of data series.

Data series	Description	Data sources
COVID-19 Index (CO)	This index was built using two indicators, that is, confirmed cases and number of death cases.	John Hopkins University of Medicine [20]
Economic support index (ES)	This index was built from 2 indicators. These include government economic support and debt / contract relief for vulnerable population. This index will be used as a proxy for the economic policy of COVID-19.	Income support, Debt or contract relief, Nov 8, 2021 [28]
Stringency index (SI)	This index was calculated from 9 indicators including workplace closures; school closures; restriction on public gathering, restriction on public events; public transport; public information campaign; stay-at-home; restrictions on national and international travel. This index will be used as a proxy for the stringent social measures of COVID-19.	Stringency Index, Nov 8, 2021 [29]
Containment & Health index (CH)	This index was calculated based on 5 indicators that represent, testing policy, contact tracing, face covering, vaccination policy and number of people vaccinated. This index will be used as a proxy for the health and containment measures of COVID-19.	Containment and Health Index, Nov 8, 2021 [30]

First, this study applied the unit root test to examine data stationarity. Most of the time series data are non-stationarity and trended in nature. The problem with non-stationary data is that standard OLS (ordinary least squares) technique provides misleading conclusions [32, 33]. Moreover, it is essential to explore the time series data for stationarity. Thus, this research used the Augmented Dickey Fuller test [34] to find the data for stationarity. This type of data is called stationary if its mean, variance, and covariance persist constant over time.

Augmented Dickey Fuller (ADF) test [34] is mostly employed to test the stationarity of the data. There are different types of equations for the ADF test, which are discussed below:

$$\Delta Y=a_{0}+\gamma Y_{t-1}+\sum_{i-i}^{p}\beta_{i}\Delta Y_{t-i}+e_{t}$$ (2)

$$\Delta Y=a_{0}+\gamma Y_{t-1}+a_{1}T+\sum_{i-i}^{p}\beta_{i}\Delta Y_{t-i}+e_{t}$$ (3)

Where *α*_*o*_ is the intercept, *γ* and ß are coefficients; and *α*_1_ shows the coefficient of the trend variable. e_t_ denotes the residual term and the summation *i* shows the length of the lags in the model that starts from *1* to *p*.

Second, this study adopted dynamic simulated Autoregressive-Distributed Lag (ARDL) model [35] to explore the policy measures of countries in ASEAN towards the reduction of the COVID-19 infection. The core objective of this paper is to comparatively analyze the responses taken by the government to minimize the spread of the corona virus. First, this study composed the COVID-19 index comprising the number of reported cases and the number of death cases according to the methodology of [31]. Thus, this study used the COVID-19 (CO) index as the dependent variable in the model. Second, this study took different policy measures adopted by governments to reduce the COVID-19 pandemic as independent variables in the model. Third, this study ensured that the dependent variable, COVID-19 Index (CO) is stationary at first difference i.e. I (1). We used the Augmented Dickey-Fuller [34] to ensure the absence of integration of the series at second difference or I(2). In addition, only one dependent variable (CO) is a potential variable for cointegration relation. The dynamic simulated ARDL model is expressed as under:

$$\Delta {\left(CO\right)}_{t}=a_{0}+{ø}_{0}{\left(CO\right)}_{t-1}+{£}_{1}{\Delta (ES)}_{t}+{ø}_{1}{\left(ES\right)}_{t-1}+{£}_{2}{\Delta (SI)}_{t}+{ø}_{2}{\left(SI\right)}_{t-1}+{£}_{3}{\Delta (CH)}_{t}+{ø}_{3}{\left(CH\right)}_{t-1}+e_{t}$$ (4)

Here the variation in the dependent variable (CO) at time (t) is a function of a constant (*a*_0_), its lagged value (*CO*)_*t*−1_); Δ(*ES*), Δ(*SI*), Δ(*CH*) at time (t), and ES, SI, and CH at lagged value; *e*_*t*_ is the residual term at time (*t*).

The ARDL bounds test approach proposed by [36] for a level relationship is examined using [37] tabulated values and p-values based on the response of the surface regression. The decision rule here is that, if the F-statistic of the joint zero estimation is greater than the upper bound critical values I(1) of all coefficients of the lagged independent variables at level and the coefficient of lagged dependent variable coefficient, then the null hypothesis of no level correlation (H_0_: ø_0_ =ø_1_ = ø_2_ = ø_3_ =0) will be rejected.

## Results and discussion

To study the characteristics of the dataset, study examines the descriptive statistics analysis presented in Table 3. These variables range from February 1, 2020, to November 8, 2021, including the COVID-19 (CO) index, economic support (ES) index, stringency index (SI) and Containment and Health index (CH). Table 4 presents the overview of statistics having the mean, median, standard deviation, Skewness and Kurtosis of the data series.

**Table 4:** Descriptive statistics of data series.

Country	Variables	Mean	Median	Std. dev.	Skewness	Kurtosis
**Brunei**	CO	0.68	0.69	1.03	2.10	4.03
	ES	54.70	54.00	1.32	1.77	1.72
	SI	44.88	49.07	11.48	-1.38	6.40
	CH	45.89	50.76	13.11	-1.56	5.43
**Cambodia**	CO	1.24	0.69	1.22	1.50	2.35
	ES	31.53	30.00	2.55	2.06	4.18
	SI	58.53	55.00	10.07	2.07	6.18
	CH	58.18	56.00	9.26	1.18	1.91
**Indonesia**	CO	8.90	9.25	1.20	-0.85	3.15
	ES	38.64	38.00	6.99	0.03	1.65
	SI	73.87	72.00	7.56	0.75	1.10
	CH	48.63	50.76	13.76	0.83	3.16
**Laos**	CO	0.13	0.00	0.39	1.17	2.04
	ES	40.01	38.00	6.56	1.40	2.59
	SI	41.99	39.00	8.88	1.31	1.75
	CH	50.69	49.00	6.96	1.09	1.24
**Malaysia**	CO	5.01	4.77	1.83	-0.35	2.72
	ES	50.20	48.00	6.95	1.45	2.32
	SI	60.43	58.00	6.97	1.19	1.39
	CH	59.97	58.00	6.49	1.42	2.78
**Myanmar**	CO	4.10	3.04	2.50	0.80	2.37
	ES	67.29	67.00	7.38	0.35	1.06
	SI	68.25	68.00	7.27	0.09	1.10
	CH	53.88	52.79	7.29	0.51	1.35
**Philippine**	CO	7.68	8.38	2.97	-1.59	4.62
	ES	55.18	54.00	6.64	0.93	0.87
	SI	65.20	64.00	7.07	1.37	2.51
	CH	50.71	49.00	7.50	1.13	1.26
**Thailand**	CO	3.49	3.43	1.33	0.67	3.82
	ES	50.04	49.00	6.59	1.08	1.43
	SI	47.41	49.00	9.42	-1.41	2.37
	CH	34.60	33.00	6.65	1.21	1.62
**Singapore**	CO	6.08	6.30	1.98	-0.43	1.90
	ES	67.99	69.76	9.48	-1.54	2.66
	SI	70.42	69.76	10.03	0.60	1.12
	CH	52.09	51.00	6.52	0.64	1.10
**Vietnam**	CO	2.49	2.64	1.40	0.21	2.38
	ES	69.36	69.33	9.90	0.63	1.37
	SI	70.43	69.00	10.65	0.84	1.38
	CH	68.70	69.00	9.64	0.86	2.08

Source: author(s) calculation

The initial stage in testing the level relationships between the COVID-19 index (explained variable) and its explanatory variables (ES, S, and CH) is to ensure that the COVID-19 index is stationarized at the first difference while independent variables can follow the property of stationarity at the level or at order one I(1). For this purpose, the ADF (Augmented Dickey-Fuller) test [34] was applied. Table 5 provides the findings of ADF unit root test. These results verified the absence of unit root problem in the data series. Consequently, all variables are either stationary at level or at first difference I(0) or I(1) except COVID-19 index (dependent variable) that is stationarized at first difference and is potential candidates for the dynamic simulated ARDL bounds co-integration.

**Table 5:** Findings of augmented dickey fuller test.

Variables		CO	ES	SI	CH
**Brunei**	Level	-1.265 (0.64)	-2.242 (0.191)	-3.126* (0.000)	-3.130** (0.024)
	1^st^ diff	-3.635* (0.005)	-4.126* (0.000)	-	-
**Cambodia**	Level	-2.428 (0.059)	-1.448 (0.559)	-1.604 (0.481)	-3.306** (0.017)
	1^st^ diff	-3.092** (0.024)	-4.968* (0.001)	-5.528* (0.000)	-
**Indonesia**	Level	-1.616 (0.137)	-2.460 (0.125)	-1.829 (0.366)	-3.619** (0.039)
	1^st^ diff	-5.273* (0.000)	-8.629* (0.001)	-4.256* (0.005)	-
**Laos**	Level	-1.342 (0.351)	-2.728 (0.069)	-1.144 (0.697)	-3.462** (0.045)
	1^st^ diff	-4.400* (0.002)	-3.876* (0.002)	-3.671** (0.044)	-
**Malaysia**	Level	-1.246 (0.329)	-3.922* (0.001)	-1.144 (0.697)	-1.422 (0.571)
	1^st^ diff	-3.035* (0.003)	-	-3.151* (0.007)	-3.520* (0.001)
**Myanmar**	Level	-2.198** (0.169)	-1.186 (0.679)	-2.665** (0.018)	-2.728 (0.069)
	1^st^ diff	-2.272** (0.019)	-2.517** (0.011)	-	-5.617* (0.001)
**Philippine**	Level	-1.671 (0.445)	-2.728** (0.039)	-3.144** (0.049)	-1.462 (0.552)
	1^st^ diff	-5.837* (0.001)	-	-	-3.422** (0.047)
**Thailand**	Level	-0.275 (0.15)	-2.331 (0.21)	-3.332* (0.006)	-2.619 (0.089)
	1^st^ diff	-4.16** (0.021)	-9.10* (0.001)	-	-5.423* (0.001)
**Singapore**	Level	-1.318 (0.628)	-3.126* (0.001)	-2.619 (0.089)	-4.130* (0.004)
	1^st^ diff	-3.035* (0.004)	-	-2.126* (0.002)	-
**Vietnam**	Level	-2.196 (0.207)	-0.665 (0.85)	-2.448** (0.027)	-0.665 (0.254)
	1^st^ diff	-2.97** (0.036)	-6.502* (0.007)	-	-2.618** (0.026)

*, ** denotes 1%, and 5% significance level; parentheses show the probability value

After fulfilling the preconditions, the author examined the cointegration relationship employing the modified bound test with KS tabulated values and estimated p-values. Series can be imbalance by the short run disruptions, but the disparity is addressed over time as the data series moves backward to a stable long-run correlation [38]. Testing the cointegration relationship is vitally important because not all data series validate the cointegration. Table 6 gives the findings of the ARDL bounds test using surface-response regression with appropriate critical values and estimated p-values [38]. The findings reveal that the values of F-calculated value is greater than upper limit values, confirmed by the statistically significant p-values. Hence, rejecting the H_o_ of no level relationship and confirms the validation of cointegration among the estimated variables.

**Table 6:** Outcome of the ARDL bounds test analysis.

	Models			1%		5%		10%		prob-value	
Series		k-values	F-statistic.	I(0)	I(1)	I(0)	I(1)	I(0)	I(1)	I(0)	I(1)
Brunei	*CO* = *f*(*ES*, *SI*, *CH*)	3	12.2**	4.29	5.61	3.23	4.35	2.72	3.77	0.02	0.01
Cambodia	*CO* = *f*(*ES*, *SI*, *CH*)	3	5.26**	4.29	5.61	3.23	4.35	2.72	3.77	0.01	0.02
Indonesia	*CO* = *f*(*ES*, *SI*, *CH*)	3	4.62*	4.29	5.61	3.23	4.35	2.72	3.77	0.01	0.00
Laos	*CO* = *f*(*ES*, *SI*, *CH*)	3	11.8**	4.29	5.61	3.23	4.35	2.72	3.77	0.02	0.00
Malaysia	*CO* = *f*(*ES*, *SI*, *CH*)	3	4.74**	4.29	5.61	3.23	4.35	2.72	3.77	0.03	0.01
Myanmar	*CO* = *f*(*ES*, *SI*, *CH*)	3	4.84*	4.29	5.61	3.23	4.35	2.72	3.77	0.01	0.00
Philippines	*CO* = *f*(*ES*, *SI*, *CH*)	3	26.8*	4.29	5.61	3.23	4.35	2.72	3.77	0.02	0.01
Thailand	*CO* = *f*(*ES*, *SI*, *CH*)	3	4.79**	4.29	5.61	3.23	4.35	2.72	3.77	0.01	0.03
Singapore	*CO* = *f*(*ES*, *SI*, *CH*)	3	5.54*	4.29	5.61	3.23	4.35	2.72	3.77	0.01	0.00
Vietnam	*CO* = *f*(*ES*, *SI*, *CH*)	3	4.84**	4.29	5.61	3.23	4.35	2.72	3.77	0.04	0.01

*, ** denote 1, and 5% level of significance.

Dynamic simulated ARDL approach is competent to calculate, predict and plot counterfactual change prediction while maintaining the stability of the explained variables with high accuracy level [38]. The stimulated dynamic ARDL adopted 5000 simulations of the vector of parameters of a multivariate normal distribution. Tables 7 and 8 present the findings of the dynamically stimulated ARDL error correction model. In Tables 7 and 8, the coefficient of *COI*_*t*−1_ for each country is significant at 1% level and carries negative sign, representing 14.9%, 24.9%, 11.1%, 45.1%, 51%, 36.6%, 37.4%, 38.2%, 39.1%, and 39.9% speed of adjusting the disequilibrium over time for Brunei, Cambodia, Indonesia, Laos, Malaysia, Myanmar, Philippines, Singapore, Thailand, and Vietnam, respectively.

**Table 7:** Findings of dynamic simulated ARDL model.

Variables	Brunei	Cambodia	Indonesia	Laos	Malaysia
*CO*_*t*−1_	-0.149 a* (0.069)	-0.249 a* (0.076)	-0.111 a* (0.042)	-0.451 a*(0.116)	-0.51 a* (0.118)
ΔES_*t*_	-0.124 ** (0.05)	-0.157** (0.058)	-0.339** (0.043)	-0.229* (0.037)	-0.56** (0.185)
ES_*t*−1_	-0.62* (0.078)	-0.422** (0.067)	-0.259** (0.05)	-0.116** (0.025)	-0.314** (0.10)
ΔSI_*t*_	-0.69** (0.109)	-0.563* (0.063)	-0.104** (0.011)	-0.337** (0.07)	-0.55* (0.178)
SI_*t*−1_	-0.374** (0.104)	-0.156** (0.036)	-0.148* (0.063)	-0.23** (0.103)	-0.313** (0.118)
ΔCH_*t*_	-0.258** (0.081)	-0.515* (0.202)	-0.815* (0.369)	-0.196** (0.049)	-0.231** (0.034)
CH_*t*−1_	-0.359** (0.09)	-0.421* (0.062)	-0.697* (0.174)	-0.473** (0.192)	-0.316** (0.155)
Constant	-0.324* (0.157)	-0.54** (0.208)	-0.341** (0.161)	-0.432** (0.182)	-0.358** (0.165)
Sims	5000	5000	5000	5000	5000
R^2^	0.75	0.73	0.98	0.71	0.79
Prob > F	0.0004*	0.0001*	0.0002*	0.000*	0.0002*

*, **, *** represent significance at 1, 5, and 10%; parenthesis () represents the standard error; ^a^ represents the speed of adjustment; Sims denotes the number of simulations.

**Table 8:** Findings of dynamic simulated ARDL model.

Variables	Myanmar	Philippine	Thailand	Singapore	Vietnam
*CO*_*t*−1_	-0.366 a* (0.167)	-0.374 a* (0.169)	-0.382 a* (0.17)	-0.391 a* (0.172)	-0.399 a* (0.174)
ΔES_*t*_	-0.407** (0.176)	-0.664** (0.238)	-0.424** (0.180)	-0.556** (0.212)	-0.44** (0.184)
ES_*t*−1_	-0.449** (0.186)	-0.457** (0.188)	-0.465** (0.19)	-0.308** (0.153)	-0.482 *(0.194)
ΔSI_*t*_	-0.49* (0.196)	-0.498** (0.198)	-0.507** (0.200)	-0.205** (0.042)	-0.523** (0.204)
SI_*t*−1_	-0.531** (0.206)	-0.333** (0.159)	-0.548** (0.21)	-0.349* (0.163)	-0.564* (0.214)
ΔCH_*t*_	-0.573** (0.216)	-0.581** (0.218)	-0.656** (0.298)	-0.763** (0.262)	-0.697** (0.300)
CH_*t*−1_	-0.763** (0.262)	-0.421* (0.062)	-0.231** (0.0343)	-0.041** (0.021)	-0.334** (0.158)
Constant	0.953** (1.43)	-0.415** (0.178)	-0.205** (0.042)	-0.804** (0.272)	-0.912* (-0.338)
Sims	5000	5000	5000	5000	5000
R^2^	0.95	0.85	0.80	0.93	0.55
Prob > F	0.000*	0.000*	0.0010*	0.0002*	0.000*

*, **, *** represent significance at 1, 5, and 10%; parenthesis () represents the standard error; a denotes the speed of adjustment; Sims denotes the number of simulations.

In Laos, the coefficient of the economic support index (ΔES_*t*_) is statistically significant at 1% significance level having negative sign in short run, while the coefficient is negative and statistically significant at 5% significance level in Brunei, Cambodia, Indonesia, Malaysia, Myanmar, Philippines, Singapore, Thailand, and Vietnam. Therefore, we accept the hypothesis that economic support measures significantly reduce the infection of the COVID-19 pandemic in these countries in the short run. Therefore, this study explored that economic support and debt / contract relief for poor population advanced by the governments play a significant role to curb COVID-19 pandemic. [39] also explored that financial support to affected developing countries is necessary so that they can fight the COVID-19. In addition, the findings concluded that, In Brunei and Vietnam, the coefficient of the stringency index (ΔSI_*t*_) is statistically significant at 1% significance level having negative sign in long-run, while the coefficient is statistically significant at 5% significance level and having negative sign in Cambodia, Indonesia, Malaysia, Myanmar, Philippines, Singapore, and Thailand. Therefore, we accept the hypothesis that the stringency measures such as workplace closures, school closures, restriction on public gathering, public transport, public information campaign, stay-at-home, restrictions on national and international travel significantly reduce the infection of COVID-19 pandemic in these countries in the long run.

In Cambodia, Malaysia, and Myanmar, the coefficient of the stringency index (ΔSI_*t*_) is statistically significant at 1% significance level with negative sign in short run, while the coefficient is negative and statistically significant at 5% significance level in Brunei, Indonesia, Laos, Philippines, Singapore, Thailand, and Vietnam. Therefore, we accept the hypothesis that the stringency measures significantly reduce the infection of COVID-19 pandemic in these countries in the short run. Moreover, the findings concluded that, in Cambodia, Malaysia, and Myanmar, the coefficient of the stringency index (ΔSI_*t*_) is statistically significant at 1% significance level with negative sign in long-run, while the coefficient is negative and statistically significant at 5% significance level Brunei, Indonesia, Laos, Philippines, Singapore, Thailand, and Vietnam. Therefore, we accept the hypothesis that the stringency measures significantly decrease the spread of COVID-19 pandemic in these countries in the long run. In addition, this research also found that the closure of workplaces, schools, restrictions on public events, closure of public transport, stay at home, restrictions on international travel, and restrictions on internal travel are necessary to reduce the infection of the COVID-19 pandemic. These findings are consistent with the results of previous studies conducted by [40]. Moreover, their findings also concluded that that quarantine and social distancing are important to minimize the infection of the COVID-19 pandemic.

In Cambodia, and Indonesia the coefficient of the Containment and Health index (ΔCH_*t*_) is statistically significant at 1% significance level with negative sign in short run, while the coefficient is negative and statistically significant at 5% significance level in Brunei, Laos, Malaysia, Myanmar, Philippines, Singapore, Thailand, and Vietnam. Therefore, we accept the hypothesis that containment and health measures such as testing policy, contact tracing, face covering, vaccination policy and number of people vaccinated play a significant role to curb COVID-19 disease in these countries in the short run. In addition, the findings concluded that, in Cambodia, Indonesia, and Philippines, the coefficient of Containment and Health index (CH_*t*_) is statistically significant at 1% significance level with negative sign in long-run, while the parameter is negative and statistically significant at 5% significance level in Brunei, Laos, Malaysia, Myanmar, Singapore, Thailand, and Vietnam. Therefore, we accept the hypothesis that containment and health measures play a vital role to curb COVID-19 pandemic in these countries in the long run. Moreover, this study found that testing policy and contact tracking, public awareness campaigns play a significant role to control the COVID-19 spread to a large extent. [41] concluded that public health preventive measures lower the percentage increase in daily COVID-19 cases. [42] also concluded that preventive health measures resulted in a stability in COVID-19 confirmed cases in Hong Kong. Government economic support for poor families, stringency, health and containment measures, must all be implemented during the pandemic to decrease the infection of COVID-19 [43].

The study employs diagnostic test (Fig 6) and explored that the residuals of the estimated models are independent. This study applied the cumulative sum test to confirm the stability of the coefficients of the models presented in (Fig 6a) to (Fig 6j). Evidence of the recursive cusum and cusum of the squares graph indicates that all the estimated variables are within the 95% confidence range, therefore, confirms that the estimated model is stable.

**Fig 6:** (a). Recursive cusum plot & cusum of squares plot for Brunei. (b). Recursive cusum plot & cusum of squares plot for Cambodia. (c). Recursive cusum plot & cusum of squares plot for Indonesia. (d). Recursive cusum plot & cusum of squares plot for Laos. (e). Recursive cusum plot & cusum of squares plot for Malaysia. (f). Recursive cusum plot & cusum of squares plot for Myanmar. (g). Recursive cusum plot & cusum of squares plot for Philippines. (h). Recursive cusum plot & cusum of squares plot for Singapore. (i). Recursive cusum plot & cusum of squares plot for Thailand. (j). Recursive cusum plot & cusum of squares plot for Vietnam.

## Conclusions

This study empirically examined various measures, including economic support and debt or contract relief measures, containment and health measures, and stringent measures implemented by ASEAN countries to reduce the spread of coronavirus in the region using a dynamic simulated Autoregressive-Distributed Lag (ARDL) approach. The study explored that government economic support and debt/contract relief program for the for the vulnerable population of COVID-19 play a vital role in the short- and long-run fight against the infection of COVID-19. In addition, the study also explored that the restriction on public events, closure of schools and workplaces, restrictions on public gathering, stay at home, closure of public transport, restrictions on domestic and international travel are essential to reduce the spread of the COVID-19 pandemic both in the short- and long-run during pandemic. Finally, this study also found that public awareness campaigns, testing policy, and social distancing also play a significant short- and long run role in minimizing the spread of the COVID-19 pandemic. Policy implications such as government economic support for vulnerable populations, schools closures, restriction on public gathering during pandemic, public awareness among the masses, and testing policy should be adopted to stop the COVID-19 spread. Protect vulnerable populations, comprising the homeless and high-density facilities such as nursing homes, prisons, hostels, retirement villages and psychiatric hospitals by monitoring and responding to their needs.

Furthermore, vaccination is essential to reduce the disease burden and mitigating future outbreaks due to the unavailability of population-level immunity to COVID-19. The results of this study imply that vaccination can have a significant impact on reducing the number of people who contract COVID-19, end up in hospital and die. There will be a huge increase in vaccine coverage and delivery capacity if existing vaccination efforts are followed by a general relaxation of all other restrictions. Despite this, our findings show that vaccines against COVID-19 have the potential to be both powerful and effective. To ensure the effectiveness of a national vaccination policy, the government must clearly communicate and use healthcare professionals as reliable sources of medical information and implement effective public health policies to address the factors responsible for the low acceptability of vaccines.

### Limitation of the study

This study excludes the country Maldives from the study due to unavailability of official data.
